# A Rapid Systematic Review of Worldwide Alcohol Use Disorders and Brief Alcohol Interventions in the Criminal Justice System

**DOI:** 10.3389/fpsyt.2022.900186

**Published:** 2022-07-07

**Authors:** Dorothy Newbury-Birch, Jennifer Ferguson, Natalie Connor, Andrew Divers, Gillian Waller

**Affiliations:** School of Social Sciences, Humanities and Law, Teesside University, Middlesbrough, United Kingdom

**Keywords:** criminal justice, offending, alcohol, brief intervention, systematic review

## Abstract

Although the relationship is complex, there is an association between alcohol use and offending behavior with an interplay between the amount drank, the pattern of drinking and individual and contextual factors. Alcohol brief interventions have been shown to be effective in primary healthcare, however there is currently a lack of compelling evidence in the criminal justice system. We carried out a rapid systematic review of the literature, which updated our review conducted in 2016. Following systematic searches, we included 36 papers on prevalence and 13 papers on effectiveness. Between 26 and 88% of individuals in the policy custody setting scored positive for an alcohol use disorder. In the magistrates court this was 95%; 31–86% in the probation setting and between 19 and 86% in the prison system. In relation to probable dependence, between 21 and 38% of individuals were shown to have probable alcohol dependence in the police custody suite setting; 39 per cent in the magistrate court system; 17–36% in the probation setting and between 18 and 48% in the prison system. This compares to 6% in the general population. We included 13 studies of effectiveness with differing outcome measures and outcomes. We conclude more studies are needed in the field to develop the current evidence base.

## Introduction

An estimated 3.8% of all global deaths and 4-6% of global disability-adjusted life-years are attributable to alcohol (1). Although the relationship is complex, there is an association between alcohol use and offending behavior (2, 3), with an interplay between the amount drank, the pattern of drinking and individual and contextual factors (4). In England and Wales, alcohol-related crime is estimated to cost society £11.4 billion (5) and drugs £20 billion annually (6). Effective interventions have the potential to significantly reduce the costs relating to substance use, as well as increase individual social welfare (7).

Hazardous drinking is a repeated pattern of drinking that increases the risk of psychological or physical problems (8), whereas harmful drinking is defined by the presence of these problems (9). Drinking at hazardous or harmful levels are often categorized as risky drinking. Previous research has shown that risky drinking is more than twice as high in the criminal justice system (CJS), in comparison with the general population, in the UK, and probable dependency up to 10 times higher (10).

Alcohol brief interventions (ABIs) are a secondary prevention activity, which are aimed at those individuals who are drinking in a pattern that is likely to be harmful to health and/or well-being. They have been frequently shown to be effective in primary healthcare (11, 12), but they are typically delivered by practitioners who are not addiction specialists, to non-treatment, opportunistic populations (13).

They largely consist of two different approaches; simple structured advice, which after screening, raises awareness through provision of personalized feedback and advice on steps to reduce drinking behavior and its adverse consequences; and an extended brief intervention, which generally involves behavior change counseling. Extended brief intervention introduces and evokes change by giving the participant the opportunity to explore their alcohol use, as well as their motivations and strategies for change. Both forms share the common aim of helping people to change drinking behavior to promote health (13).

There is a wide variation in the duration and frequency of ABIs. However, typically they consist of between one and four sessions and are very short in nature (between five and 60 minutes) (14). They generally include personalized feedback on alcohol intake in relation to what the recommended limits are, discussion of both health and social risks and may include setting personal targets which can include psychological and motivational interviewing (14). One example of this is using the FRAMES (feedback, responsibility, advice, menus, empathy, self-efficacy approach (13).

They are generally delivered in an opportunistic way by practitioners other than addiction specialists, in a wide variety of settings (12). Due to the established links between risky drinking and crime and the costs to society, in both health and social care, it is important to find interventions that are effective. It has been shown that interventions that capitalize on the “teachable moment” are conducive with behavior change, where individuals consider their alcohol use within the context of their offending behavior and its punitive consequences (15, 16). However, to date, there is a dearth of evidence relating to alcohol use disorders (AUDs) and the use of brief interventions in the CJS (10, 17). Therefore, this review was proposed as a way to update and collate the evidence around the prevalence of AUDs within the CJS and to review the evidence around the efficacy of alcohol brief interventions within these populations.

## Aim

The aim of this rapid review was to update our 2016 review (10) and to identify the levels of AUDs in the various stages of the CJS around the world. Secondly it aimed to narratively review worldwide studies of the effectiveness of ABIs in the various stages of the CJS.

## Methods

We carried out a review of the international literature, employing the Preferred Reporting Items for Systematic reviews and Meta-Analyses (PRISMA) guidelines, which ensure comprehensive reporting within systematic reviews (18). This rapid systematic review was conducted to update the review undertaken in 2016 (10). However, the original review only included prevalence in the UK, whereas this current review was extended to include worldwide literature.

### Inclusion Criteria

Any language paper was eligible for inclusion.

Papers were included in the review if they contained information around alcohol use prevalence or were trials investigating the efficacy of ABIs, within the CJS. The following criteria were used for selection;

#### Alcohol Use Prevalence

This review sought to identify the prevalence of AUDs in the CJS worldwide, by searching the available evidence. To ensure reliability, it was important for papers to use a screening tool that is validated when assessing the prevalence of AUDs (10). Therefore, we included papers that employed the use of the Alcohol Use Disorders Identification Test (AUDIT), which is considered to be the gold standard of tools used to identify AUDs in healthcare settings (19). The AUDIT gives prevalence data and is not a diagnostic tool.

The 10 question AUDIT is scored between 0–40. A score of 8+ for adults indicates an alcohol use disorder; 8–15 indicates hazardous drinking, 16–19 harmful drinking and a score of 20+ indicates probable dependence (20). It has been shown to have 92% sensitivity and 94% specificity (20). Furthermore, it has been shown to be effective in the various stages of the CJS (21). Any papers that did not report the use of the AUDIT, to identify prevalence, were excluded.

#### Alcohol Brief Interventions

Using the same literature searches we also looked to include trials of ABIs in the CJS. We used the definitions of ABIs as listed in the background and sought to include studies with control groups comprising of any other intervention, no assessment, assessment only, information only or treatment as usual. We included studies that included psychosocial interventions up to a total of 3 hours of ABIs either in one or multiple sessions.

### Exclusion Criteria

Papers predating 2000 were not considered, and searches were restricted to 2000- present (January 2022). We also excluded papers that included a drug and alcohol intervention where alcohol information could not be easily extracted.

#### Searches

The following databases; EBSCO (Child Development & Adolescent Studies, CINAHL Complete, Criminal Justice Abstracts with Full Text, MEDLINE, APA PsycArticles, Psychology and Behavioral Sciences Collection, APA PsycInfo) and Scopus were searched using the search terms alcohol, screening, crime, police probation, court, jail, prison and variations of these in the title, keywords and abstract.

Two authors were involved in the sifting of the published papers (DNB and JF). DNB reviewed all abstracts and full papers and JF acted as the second reviewer, reviewing 20% to ascertain that all decisions matched, which they did, without the need for a third reviewer. Endnote was used to manage the data in the sifting stages, whilst data extraction was carried out using Microsoft Excel, which was again undertaken by DNB and JF reviewing 20%. Data was extracted in the same way as our previous review, using the same data extraction tables, except that the country of study was added to the prevalence extraction table (10).

Gray literature was also searched from around the world, with variations of the search terms being entered into Google and the first 300 hits were investigated by NC, AD and GW. We also interrogated our previous papers on the subject (10, 17), screened the reference lists of included papers and reached out through the International Network on Brief Interventions for Alcohol and Other Drugs (Inebria- http://inebria.net/) and Twitter to obtain any further articles, and to ensure no potentially relevant studies had been overlooked.

#### Quality Assessment

The relevant screening tools from the Critical Appraisal Skills Programme (CASP) were used to quality assess any included papers (22). The QA was carried out across the research team (GW, AD and NC) with 20% being double checked. High risk of bias was recorded if “no” or “unsure” was recorded for 6 or more of the 11 questions on the tool. Medium risk of bias was assigned if “no” or “unsure” was recorded for 4–5 questions and Low risk for 1–3 questions, as in our previous study (17).

## Results

In total 10,898 papers were identified from the initial searches. Following the first sift, 189 full papers were assessed for inclusion. After completion of full text screening 40 papers were deemed eligible for inclusion. Figure 1 provides a breakdown of the numbers of papers and gray literature excluded at each stage and how many papers were used in assessing the prevalence vs. the alcohol brief intervention efficacy.

**Figure 1:** Data flow.

## Results—Prevelance—Adults

In total, 39 studies from 34 papers were included, as presented in Table 1. The majority of papers were from the UK (4, 11, 21, 23, 24, 26–32, 34–37, 39, 41–43, 47–49, 54), two from Sweden (25, 44) and one each from Australia (51), Brazil (45), Ethiopia (52), France (40), Holland (38), Norway (50), Ukraine (46) and the USA (53).

**Table 1:** Alcohol use disorder prevalence.

**References**	**Country**	**% m/f (total *n*)**	**Age**	**AUD positive**	**AUD ranges**	**QA**
**Police custody suits**						
Hopkins and Sparrow (23)	England	89% male (*n =* 805)	Mea*n =* 27	88%	PD = 35%	LR
Brown et al. (24)	England	81% male (*n =* 229)	29.4 ± 11	76%	None given	LR
Durbeej et al. (25)	Sweden	91% male (*n =* 181)	33 ± 10.9	14.66+10.19	None given	LR
Tobutt and Milani (26)	England	92% male (*n =* 12)	18+	14.9 ± 1.4	None given	HR
Barton (27)	England	85% male (*n =* 3,900)	17+	64%	Haz = 32%; Harm = 11%; PD = 21%	LR
Mccracken et al. (28)	England	86% male (*n =* 4,739)	18+	85%	Haz = 36%; Harm = 13%; PD = 37%	MR
Kennedy et al. (29)	England	83% male (*n =* 2,177)	18+	84%	Haz = 38%; Harm = 11%; PD = 38%	MR
Addison et al. (30)	England	not given (*n =* 720)	18+	54%	None given	LR
Samele et al. (31)	England	93% male (*n =* 134)	31.2 ± 10.4	26%	None given	LR
**Magistrates court**						
Watt et al. (32)	Wales	100% male (*n =* 262)	I: 23.6 ± 4.7 C: 22.8 ± 4.6	95%	PD = 39%	LR
**Probation**						
MacAskill et al. (33)	Scotland	100% male (*n =* 216)	18–64	73%	Haz 27%; Harm = 9%; PD = 36%	LR
Newbury-Birch et al. (34)	England	86% male (*n =* 262)	18+	M = 69% F = 53%	M-Haz = 26%; M-Harm *n =* 11%; M-PD = 35%. F-Haz = 25%; F-Harm = 3%; F-PD = 25%	LR
Newbury-Birch et al. (35)	England	85% male (*n =* 525)	31 ± 10.9	86%	Haz = 43%; Harm/Dep = 42%	LR
Pluck et al. (36)	England	87% male (*n =* 173)	36.0 ± 13.5	11.6 ± 10.7	PD = 23%	LR
Orr et al. (37)	Scotland	85% male (*n =* 195)	Mea*n =* 31	59%	PD = 17%	MR
Hildebrand and Noteborn (38)	Holland	86% male (*n =* 371)	not given	M = 47% F = 20%	M-PD = 12%; F-PD = 5%	LR
Fitton et al. (11)	England	100% male (*n =* 32)	58.1 ± 6.9	31%	mean AUDIT 7.2 ± 8.5	HR
**Prison**						
Lader et al. (39)	England and Wales	Remand: 92% male (*n =* 339)	16+	M = 62%; F = 13%	M-Haz = 28%; M-Harm/PD = 33%. F-Haz = 5%; M-Harm/PD = 8%	MR
Lader et al. (39)	England and Wales	Sentenced: 68% male (*n =* 250)	16+	M = 70%; F = 51%	M-Haz = 34%; M-Harm/PD = 36%. F-Haz = 25%; M-Harm/PD = 25%	MR
Maggia et al. (40)	France	100% male (*n =* 47)	27.3 ±8	19%	None given	LR
McMurran and Cusens (41)	England	100% male (*n =* 126)	30.52 ± 10	86%	None given	MR
Newbury-Birch et al. (34)	England	94% male (*n =* 411)	18+	M = 59%; F = 63%	M-Haz = 19%; M-Harm = 4%; M-PD = 36%. F-Haz = 21%; F-Harm = 0; F-PD = 42%	LR
Begun et al. (42)	England	100% female (*n =* 1,181)	18+	67%	None given	MR
Parkes et al. (43)	Scotland	Remand: 100% male (*n =* 137)	Median *=* 27	68%	Haz = 24%; Harm = 10%; PD = 34%	MR
Parkes et al. (43)	Scotland	Sentenced: 100% male (*n =* 122)	Median *=* 27	83%	Haz = 31%; Harm = 9%; PD = 39%	MR
Graham et al. (4)	Scotland	100% male (*n =* 96)	18+	73%	Haz = 25%; Harm = 43%; PD = 43%	LR
Konstenius et al. (44)	Sweden	100% female (*n =* 96)	39.7	33%	21% 6–17 on AUDIT; 22% >18 on AUDIT	LR
Nunes et al. (45)	Brazil	100% female (*n =* 178)	34.2 ± 9.6	7.25 ± 10.6	None given	LR
Azbel et al. (46)	Ukraine	80% male (*n =* 402)	31.9	57%	None given	LR
Kissell et al. (47)	England	100% male (*n =* 242)	26.5	81%	PD = 48%	MR
Wainwright et al. (48)	England and Wales	100% male (*n =* 105)	42 ± 14	56%	Mean 13.87 ± 12.10	LR
Holloway et al. (49)	England and Scotland	100% male (*n =* 502)	33 ± 10	80% sentenced; 82% remand	PD 34% sentenced and 49% remand	LR
Pape et al. (50)	Norway	94% male (*n =* 1,446)	not given	55%	PD = 18%	LR
Kerslake et al. (51)	Australia	91% male (*n =* 371)	34.1 ± 9.3	35%	None given	LR
Haile et al. (52)	Ethiopia	100% male (*n =* 347)	27.8 ± 11.4	59%	PD = 21%	LR
**Police, probation and prison together**						
Coulton et al. (21)	England	57% male (*n =* 205)	31.1 ± 9.9	73%	Haz:26%; harm/DP = 75%	LR
**Young people**						
Thayer et al. (53)	USA	80% male (*n =* 125)	16.6 ± 1.1	59% (4+)	None given	LR
Newbury-Birch et al. (54)	England	85% male YOT/prison (*n =* 411)	11 to 17	64% (8+)	Haz = 22%; Harm = 12%; PD = 30%	LR
Newbury-Birch et al. (54)	England	85% male YOT/prison (*n =* 411)	11 to 17	81% (2+)	PD = 77%	LR

*M, male; F, female; AUD, positive on screening tool for an alcohol use disorder; Haz, hazardous drinking; Harm, harmful drinking; PD, probably dependent; LR, low risk of bias; MR, medium risk of bias, QA, Quality assessment*.

### Police, Probation and Prison Together

One study of low risk from England included participants from the police, probation and prison together (21). The study included 205 participants and showed that 73% had an AUD with 26% as hazardous drinkers and 75% harmful or possibly dependent.

### Police Custody Suites

Nine studies were found relating to the police custody suite setting (23–31). Six studies were classified as low risk (23–25, 30, 31), two as medium risk (28, 29) and one as high risk (26). Eight were conducted in England and one in Sweden (25) and included 12,897 participants (range 12–4,739) and the majority of participants were male (Table 1).

Two of the studies gave mean AUDIT scores 14.7 ± 10.19 and 14.66 ± 10.19 (25, 26). The prevalence of AUDIT positives ranged from 26 to 88% with the median being 76%. Four studies reported prevalence of probable dependence (23, 27–29). These ranged from 21 to 38% (Table 1).

### Magistrates Court

One study was found (low risk) in relation to prevalence amongst those at a magistrates' court in Wales (32). Of those screened 95% scored positive for an AUD (8+ on AUDIT) and 39% as being probably dependent (20+ on AUDIT). The eligibility for the study, however, was that the participant had been sentenced for a violent crime committed whilst intoxicated. This would, in part, explain the high prevalence rates (Table 1).

### Probation

Seven studies were found in the probation setting (11, 33–38). Five were classified as low risk (33–36, 38), one medium risk (37) and one high risk (11). Four were conducted in England) (11, 34–36), two in Scotland (33, 37) and one in Holland (38) and included 1,774 participants (range 32–525) and the majority of participants were male (Table 1). Two studies gave mean AUDIT scores: 11.6 ± 10.7 and 7.2 ± 8.5 (36, 38). Prevalence rates for an AUD ranged from 31 to 86% and probable dependence between 5 and 36%. Two studies gave prevalence rates for women; AUDIT positive 20 and 53%, probable dependence was 25 and 5% (34, 38).

### Prison

We found 18 studies from 16 articles (4, 34, 39–46, 48–50, 52, 53). Eleven studies were low risk (4, 34, 40, 44–46, 48–52) with the rest classified as medium risk (39, 41, 42, 47).

Of the 15 articles, four were conducted in England (34, 41, 42, 47), two in England and Wales (39, 48), two in Scotland (4, 43), one each in England and Scotland (55), France (40), Ukraine (46), Sweden (44), Brazil (45), Norway (50), Ethiopia (52) and Australia (56). The studies included 6,398 participants (range 47–1,446) (Table 1).

Two of the studies gave mean AUDIT scores 7.25 ± 10.6 and 13.87 ± 12.10 (45, 48). Three studies gave prevalence rates for women (13; 51 and 63%) (34, 39). In the same studies probable dependence for women was shown as 8, 25 and 42%. AUDIT positive rates in all studies ranged from 19–86% and probable dependence from 21 to 48% (Table 1).

### Young People

Three studies from two papers of low risk were included (53, 54). One article was conducted in England (54) one in the USA (53). The studies included 536 participants (range 125–227).

Thayer et al. (53) conducted a study in juvenile justice diversion in the USA and found that 59% of the population scored 4+ on the AUDIT. Newbury-Birch et al. (35) carried out a study with young people aged 11–17 in Youth Offending Teams (YOTs) and young offenders' institutions (prison) in England. They found that when using adult cut-offs on the AUDIT (8+) 64% scored positive for an AUD. When using the cut off of 2+ on AUDIT recommended by Knight et al. (57) the majority of young people (81%) scored positive for an AUD.

## Results—Interventions

In total, 13 studies were included (Tables 2, 3). Seven studies were from the UK (26, 28–30, 32, 34, 37) and six from the USA (42, 56, 58–61).

**Table 2:** Details of included papers.

**References**	**Age (ethnicity) (% male)**	**Follow-up period (follow up rates)**	**Alcohol screening used and cut-off used (who screened)**	**Intervention (number randomized)**	**Control (number randomized)**	**QA**
**Custody suites**						
Tobutt and Milani, (26) (England)	MIBI: mean 25 ± 3.86; BI: 32.43 ± 7.9 (75% White British, 17% Pakistani, 8% mixed race) (92% male)	12 weeks (100%)	AUDIT 8–19 (arrest referral worker)	MIBI (no information given) (*n =* 5) or BI (no information given) (*n =* 7)	Not applicable	MR
Kennedy et al. (29) (England)	>90% white	6 months (7%)	AUDIT 8+ (various practitioners)	Various brief interventions (20–120 min) (*n =* 2,177)	Matched control group (*n =* 2,177)	HR
McCracken et al. (28) (England)	93% white	12 months (100%)	AUDIT 8+ (various practitioners)	Various brief interventions (20–120 min) (*n =* 4,739)	Matched control group (*n =* 4,711)	HR
Addison et al. (30) (England)	Mean 32.47 ± 10.96 (94% White British) (83%)	6 and 12 months (25, 23%)	AUDIT 8+ (Detention Officer)	1: Structured brief advice (5 min) (*n =* 165); 2: Structured brief advice (5 min) and brief lifestyle counseling (20 min) (*n =* 61)	Client information leaflet (*n =* 79)	LR
**Magistrates court**						
Watt et al. (32) (Wales)	I: 23.6 ± 4.7 (92.4% White; 3.8% Black; 3.8 other) (100%) C: 22.8 ± 4.6 (93.9% White; 2.3 Black; 3.8% other) (100%)	3 and 12 months (87, 75%)	AUDIT 8+ (Researcher)	1 session of MI (15–20 min) (*n =* 135)	TAU (*n =* 134)	LR
**Probation**						
Newbury-Birch et al. (35) (England)	Mean 31.0+10.9 (White 76%) (85%)	6 and 12 months (68, 60%)	AUDIT 8+ (Offender Managers)	1: Structured brief advice (5 min) (*n =* 178); 2: Structured brief advice (5 min) and brief lifestyle counseling (20 min) (*n =* 163)	Client Information leaflet (*n =* 184)	LR
Orr et al. (37) (Scotland)	18+ no other information for the RCT	6 and 12 months (13, 7%)	AUDIT 8–19 (Community justice staff)	BI (no information) (*n =* 43)	Screening and feedback (*n =* 39)	HR
**Prison**						
Davis et al. (58) (USA)	Mean 45.7 ± 7.7 (49% Caucasian; 38% African-American) (97% male)	2 months (41%)	Form-90 alcohol tool (researcher)	1 session of MI (60 min) (*n =* 36)	TAU and information on local services (*n =* 37)	HR
Stein et al. (59) (USA)	Mean 34.1 ± 8.9 (71% Caucasian; 19% African-American; 7% Hispanic) (100% female)	1, 3 and 6 months (76, 79, 79%)	AUDIT 8+ (researcher)	2 sessions of MI (45–60 min): 2nd session 1st follow = up (*n =* 125)	TAU (*n =* 120)	LR
Begun et al. (42) (USA)	Mean 35.7 ± 8.7 (57% African-American; 31% White; 6% Hispanic) (100% female)	2 months post release (20%)	AUDIT-12 8+ (researcher)	1 session of MI (60–90 min) (*n =* 468)	TAU (*n =* 261)	MR
Owens et al. (60) (USA)	Mean age 34.4 ± 9.8 (27.5% Hispanic; 20% Native American/Alaskan Native; 17.5% African American; 7.5% Biracial/multiracial/other) (100% male)	Between 1 and 3 months (63%)	ASSIST (Researcher)	1 session of MI (50–60 min) (*n =* 23)	1 session of educational videos (50–60 min) (*n =* 17)	MR
**Young people**						
Stein, Clair et al. (56) (USA)	Mean 17.1 ± 1.1 (33% White; 29% Hispanic; 28% African-American) (86% male)	3 months (86%)	Risk and Consequences Questionnaire- Alcohol (Researcher)	2 sessions of MI (1 = 90 min; 2 = 60 min) (*n =* 189 randomized, no breakdown given)	2 sessions of relaxation training (1 = 90 min; 2 = 60 min)	LR
Stein, Lebeau et al. (61) (USA)	Mean 17.1 ± 1.1(32% Hispanic; 30% African-American; 30% White) (84% male)					LR

*MI, Motivational Interviewing; min, minutes; TAU, Treatment as Usual*.

**Table 3:** Outcome measures and significant results of included studies.

**References**	**Outcomes (measures)**	**Significant results**
Tobutt and Milani, (26)	P: Mean AUDIT score S: Illicit drug use S: Money spent on alcohol S: Number of arrests S: Arrest type	No significant results related to alcohol.
Kennedy et al. (29)	AUDIT compared to Alcohol Intervention records General Health Questionnaire Arrest data	No significant results related to alcohol.
McCracken et al. (28)	Arrest data	No significant results related to alcohol.
Addison et al. (30)	P: eligible participants P: % followed-up S: AUDIT range S: Readiness to change (RTQ) S: Quality of life (EDQ-5-L) S: Arrest data	No significant results related to alcohol.
**Magistrates court**		
Watt et al. (32)	AUDIT 7 day drinking diary Illicit substance use Readiness to change (RTQ) Injury Recidivism rates	Injury was significantly less for those who had received the intervention (27.4%) than those who had not (39.6%; CI = −0.23, −0.009). At 3-month follow-up, significantly more participants in the intervention group (31%; *n =* 37) than control group (16%; *n =* 18) demonstrated an increase in their readiness to change drinking behavior (χ2 = 8.56; df = 2; P = 0.014), but this did not persist at 12-month follow-up.
**Probation**		
Newbury-Birch et al. (35)	P: 8+ on AUDIT S: Quality of life (EQ-5D) S: Readiness to change (RTQ) S: Patient Satisfaction S: Service Use S: Recidivism rates	OR of receiving a conviction was significantly lower in the brief advice (OR = 0.50; 95% CI = 0.33–0.80) and brief lifestyle counseling (OR = 0.54; 95% CI = 0.33–0.89) groups compared with the client information leaflet group.
Orr et al. (37)	AUDIT	No significant results related to alcohol.
**Prison**		
Davis et al. (58)	P: Engagement with services with VA substance abuse services (TSR) S: Contact with other substance abuse services (TSR) S: substance use (Form 90) S: Consequences (SIP) S; Addiction Severity (ASI) S: Readiness to change (RTC)	Those in the IG were statistically more likely to schedule appointments at both VA services with 60 days (66.7 vs. 41%; *p* = 0.025).
Stein et al. (59)	Drinking diary; Alcohol use disorders (AUDIT)	Intervention effects on abstinent days were statistically significant at 3 months (odds ratio = 1.96, 95% CI 1.17, 3.30).
Begun et al. (42)	P: Engagement with substance abuse treatment services P: Level of reported alcohol use (AUDIT-12)	Mean reduction in AUDIT score from baseline to follow-up were greater in the intervention group [F (1,148) = 6.336, *p* ≤ 0.001].
Owens et al. (60)	Feasibility Pre-intervention motivation and confidence ratings IDPA to assess social networks ASI criminal and treatment history Alcohol and substance use Form-90	No significant results related to alcohol.
**Young people**		
Stein, Clair et al. (56)	Risk and consequences of drinking (RCQ-A) Depression (CES-D)	No significant results related to alcohol.
Stein, Lebeau et al. (61)	Alcohol and drug use (structured clinical interview for DSM-IV) Depression (CES-D) Alcohol use (TLFB)	No significant results related to alcohol.

*P, Primary outcome; S, Secondary outcome; IG, Intervention Group; CG, Control Group; ASI, Addiction Severity Index; RSQ-A, Risks and Consequence Questionnaire – Alcohol; TSR, Treatment Services Review; SIP, Short Inventory of Problems; DSM-IV, Diagnostic and Statistical Manual of Mental Disorders, 4th. Edition; CES-D, Center for Epidemiological Studies - Depression; TLFB, Time Line Follow Back; AUDIT, Alcohol Use Disorders Identification Test; VA, Veterans Association; RTQ, Readiness to Change Questionnaire; EQ-5D Euroqol Quality of Life; OR, Odds Ratio*.

### Custody Suite

Four studies were found in relation to the custody suite (26, 28–30). Two of the studies were from different phases of the same study (28, 29). All were from England. Three were high risk (26, 28, 29) and one low risk (30) (Tables 2, 3).

#### Focus

A scheme to deliver brief interventions (<30 min) in custody suites after the arrest, or in a non-custody venue, was carried out across 12 police forces in the UK between 2007 and 2010 in two phases (28, 29). Both phases used a matched control group and looked at arrest data differences. Addison et al. (30) carried out a pilot feasibility study of brief interventions in police custody suites and compared two interventions to control condition of feedback and a leaflet with a six and 12 month follow-up period. Tobutt and Milani (26) carried out a small study (*n* = 12) of motivational interviewing and brief intervention. They did not give information on what the intervention involved. All were followed up at 12 weeks.

#### Effect

No statistically significant differences were found in any of the studies (26, 28–30).

### Magistrates Court

One study (low risk) was found for the magistrates' court setting (32).

#### Focus

Randomized Control Trial (RCT) that compared a control condition of usual care (*n* = 134) to a single 15–20-min manualised session of brief intervention (*n* = 135) in a magistrates' court in Wales, UK. The interventions were based on the work of Miller and Rollnick (13).

#### Effect

No significant findings were found in any of the alcohol use measures (AUDIT, total number of standard weekly drinks or number of drinking days) or recidivism. Injury was significantly less for those who had received the intervention (27.4%) than those who had not (39.6%; CI = −0.23, −0.009). At 3-month follow-up, significantly more participants in the intervention group (31%; *n* = 37) than control group (16%; *n* = 18) demonstrated an increase in their readiness to change drinking behavior (χ2 = 8.56; df = 2; *P* = 0.014), but this did not persist at 12-month follow-up.

### Probation

Two studies were found in the probation setting. Both were from the UK (35, 37). Newbury-Birch et al. (35) had a low risk of bias and Orr et al. (37) a high risk of bias.

#### Focus

A pilot RCT with offenders on probation on community service orders was carried out in Scotland (37). In total, 82 offenders were randomized (no information on randomization group was given for 11 offenders). A pragmatic cluster RCT of the effectiveness of two different brief intervention strategies compared to a control condition of feedback on AUDIT score and an information leaflet at reducing risky drinking in the probation setting in England (35). Probation offender managers were recruited across three areas of England (the North East, South East and London). They were randomized to one of the three conditions—each of which built upon the previous one; feedback on screening outcome and a client information leaflet control group, 5 min of structured brief advice, and 20 min of brief lifestyle counseling.

#### Effect

No effectiveness data was available in the Orr et al. (37) study as they only followed 22% of participants up (37). In the Newbury-Birch study 68 and 60% of participants were followed up at 6 and 12 months respectively (35). No significant differences between groups were found in relation to AUDIT status. Those in the brief advice and brief lifestyle counseling intervention groups were statistically significantly less likely to reoffend (36 and 38%, respectively) than those in the information leaflet group (50%) in the year following intervention (35).

### Prison

Four studies from the USA were found for the prison system (42, 58–60). One was assessed as low risk (59), two as medium risk (42, 60) and one as high risk (58).

#### Focus

Davis et al. (58) carried out an RCT of veterans in a USA county jail. Participants were recruited in the month prior to leaving jail. Despite various attempts to contact people at the two-month follow-up period, only 41% of participants were followed up. An RCT to evaluate brief intervention for alcohol use and risky sexual behavior among women in a prison in the USA was carried out by Stein et al. (59). Women were eligible for the trial if they had consumed alcohol at a hazardous level (four or more drinks on at least three occasions in the previous 3 months or identified as a hazardous drinker in the past year using the AUDIT) and if they had recently engaged in risky sexual behavior. The first session of motivational interviewing was delivered in prison with the second taking place approximately one to three months after leaving prison. Participants were followed up at 3 and 6 months. Owens and McCrady (60) carried out a pilot RCT with adult males in a large detention center in the USA with individuals who were drinking at a moderate or high level in the 12 months prior to incarceration. The two conditions both had active ingredients. Participants were randomized to either take part in a 50–60 min in-person motivational interview intervention or were asked to watch two educational videos. Participants were followed up at 3 months post intervention.

#### Effect

In the Davis et al. (58) study no differences were found between groups for any alcohol measures. Those in the intervention group were more likely to schedule appointments at a veterans' addiction clinic following their release (67 vs. 41%; *p* < 0.03) (58). Stein et al. (59) found motivational interview intervention effects on abstinent days was statistically significant at 3 months (OR = 1.96, 95% CI 1.17,3.30). Although, this effect was not maintained at 6-month follow-up. There was no significant difference between participant groups for the number of drinks consumed per drinking day. The study suggests that brief motivational interviewing may be effective at reducing the frequency of alcohol use in the short term but further sessions may be necessary to maintain the effect in the longer term. Begun et al. (42) found a mean reduction in AUDIT score greater in intervention group [F (1,148) = 6.336, *p* ≤ 0.001. Owens and McCrady (60) did not find any statistical differences and because of a low-response rate (20%) Begun et al. (42) could not test any effectiveness of the intervention.

### Young People

Two studies with a low risk of bias were found from the USA from the same author (56, 61).

#### Focus

Comparison of two sessions of motivational interviewing compared to relaxation therapy for young people in juvenile correctional facilities (56, 61). The studies were designed to evaluate the effective of depression on reducing alcohol and marijuana use.

#### Effect

Stein, Clair et al. (56) did not find any significant effects between group however Stein, Lebeau et al. (61) found that those in the motivational interview group reported a significantly lower average number of drinks consumed per day, a lower prevalence of heavy drinking days and a lower percentage of days that more than five drinks were drank at three months post-release. Participants were also automatically enrolled into a substance misuse programme which involved 2 h per week of psycho-education for alcohol and drug use for a period of 8 weeks. It is unclear if and how this contributed to the results (61).

## Discussion

In the prevalence section 39 studies (36 papers) were included. The majority of papers were from the UK (4, 11, 21, 23, 24, 26–32, 34–37, 39, 41–43, 47–49, 54), two from Sweden (25, 44) and one each from Australia (51), Brazil (45), Ethiopia (52), France (40), Holland (38), Norway (50), Ukraine (46) and the USA (53).

Using the AUDIT screening tool on the whole samples, between 26 and 88% of individuals in the policy custody setting scored positive for an AUD. In the magistrates court this was 95%; 31–86% in the probation setting and between 19 and 86% in the prison system. In relation to probable dependence, between 21 and 38% of individuals were shown to have probable alcohol dependence in the police custody suite setting; 39 per cent in the magistrate court system; 17–36 % in the probation setting and between 18 and 48% in the prison system. This compares to 6% in the general population (62). Furthermore, for young people, levels of AUD, using the adult cut-off on AUDIT, are high (64%) and levels of probable dependence were also high (30%). We found levels high across the world in the CJS and indicates similarity across different points of the CJS.

In the efficacy section we included 13 studies which was three more than in our 2016 review (10), however this still shows a scarcity of studies in this area. There are a number of reasons why this may be, including “how to measure alcohol consumption when someone has been in prison for a period of time” and the ethical arrangements needed for carrying out research in the CJS (10).

Although the evidence base relating to prevalence rates of AUDS in the CJS globally is increasing, there is still very little evidence of efficacy or effectiveness in the CJS and because there are so few studies it is impossible to assess fully withing different settings in the CJS. Since our last review, we were only able to identify three more published studies, with the majority of studies coming from the USA. This is primarily because of the issues related to when and how you measure alcohol consumption, when someone is incarcerated for a long period of time. Although there are some promising findings within the included studies, we believe more robust evidence is needed in relation to all of the stages in the CJS.

Similarly to healthcare settings, the lack of available evidence in the CJS can be attributed to issues such as workload and the time needed to undertake robust studies (10, 24, 35, 63). More work is also needed around identifying who the best people, in each of the CJS, are to deliver alcohol screening and brief interventions. Another of the main issues experienced when conducting trials in the CJS is being able to successfully follow up participants. This is in large due to the population being “hard to reach” and often falling victim to their chaotic lifestyles (37).

We found, as other studies have (10, 17), that studies examining the effectiveness of risky drinking interventions are still scarce. Another challenge associated with conducting research in the CJS is the necessity of using self-report follow-up data (10, 17, 64). Another fundamental issue is that studies include different measurement tools and outcomes, with outcomes decided upon based on the research funding. We have recently published a Core Outcome Set for Alcohol Brief Interventions to improve the measurement of alcohol-related change (65–67) which will help researchers use the same measurements in studies of brief interventions in the future. Another concern is the differences found in different studies on the active ingredients of different control groups which is an issue that effects both health and criminal justice research (35, 68, 69).

As research moves forward, it could be argued that the stages in the CJS described above are analogous to the health care system. Police stations are busy and chaotic, much like accident and emergency departments. Probation is similar to primary care, appointments made and an emphasis on dealing with the underlying issues, whereas prison is similar to hospital wards in as much as often the person is there for a period of time (10, 17). This information and analogy can help us identify key strengths and weaknesses that can be learned in these settings.

## Conclusion

This present study shows that levels of AUDs and probable dependence are high across all stages of the CJS. We need more robust research studies across all stages of the CJS in order to ascertain efficacy of alcohol screening and brief interventions.

## Data Availability Statement

The original contributions presented in the study are included in the article/supplementary material, further inquiries can be directed to the corresponding author.

## Author Contributions

DN-B wrote the first draft of the article. All authors contributed to the final article, design, and the carrying out of the systematic review. All authors contributed to the article and approved the submitted version.

## Conflict of Interest

The authors declare that the research was conducted in the absence of any commercial or financial relationships that could be construed as a potential conflict of interest.

## Publisher's Note

All claims expressed in this article are solely those of the authors and do not necessarily represent those of their affiliated organizations, or those of the publisher, the editors and the reviewers. Any product that may be evaluated in this article, or claim that may be made by its manufacturer, is not guaranteed or endorsed by the publisher.
